# Exact Solutions of Three Types of Conformable Fractional-Order Partial Differential Equations

This article has been retracted.

**DOI:** 10.1155/2022/5295115

**Published:** 2022-07-30

**Authors:** Lijun Ma

**Affiliations:** School of Science, Hebei University of Technology, Tianjin 300401, China

## Abstract

Fractional calculus is widely used in biology, control systems, and engineering, so it has been highly valued by scientists. Fractional differential equations are considered an important mathematical model that is widely used in science and technology to describe physical phenomena more accurately in terms of time memory and spatial interactions. The study of exact solutions of fractional differential equations helps to understand these complex physical phenomena and dynamic processes. The results show that the method is simple and clear. In addition, with the help of MAPL, we provide some 3D maps with accurate solutions.

## 1. Introduction

The mathematical models of many problems in life can eventually be transformed into solving integer differential equations. The development of integer integral is relatively complete from both theoretical analysis and numerical solution [1]. Fractional calculus is widely used in biology, control system, and engineering, so it has been highly valued by scientists [2]. Fractional derivatives, mainly including Caputo derivative, Riemann–Liouville derivative, and Hadamard derivative, are determined by singular integral and calculated by more complex methods [3]. The properties of conformal fractional derivative are studied. It is found that it has many properties of classical integral. Some of them were selected using MAPL and their 3D images are shown. Furthermore, we observe that this simple and easy method is an effective method for solving the fractional co-movable differential equation.

Through extensive literature search, we found that fractional-order differential equations in Banach space have received a lot of attention from many scholars, especially the review of finite dimensional fractional-order differential equations and their contained edge value problems by famous foreign scholars [6], which has guided the direction for the in-depth study. Liu et al. [7] discussed the following conformable fractional-order differential equation side value problems:

(1) $$\begin{array}{c} \left\{\begin{array}{c} T_{\alpha }y\left(t\right)+f\left(t,y\left(t\right)\right)=0,\\ y\left(0\right)=0,y\left(1\right)=\lambda \int_{0}^{1}y\left(t\right)\text{d}t. \end{array}\right.\;t\in J≔\left[0,1\right], \end{array}$$

*T*_*α*_ is a continuous function of “conformable fractional-order derivatives”, 1 < *α* < 2 < *f* : *J* × *R*^+^⟶*R*^+^.

Inspired by the above paper, this paper focuses on the Banach space with conformable fractional-order edge value problem (BVP):

(2) $$\begin{array}{c} \left\{\begin{array}{c} T_{\alpha }u\left(t\right)=f\left(t,u\left(t\right)\right),\\ u\left(0\right)=\int_{0}^{T}g\left(s,u\left(s\right)\right)\text{d}s,u\left(T\right)=\int_{0}^{T}h\left(s,u\left(s\right)\right)\text{d}s. \end{array}\right.\;t\in J≔\left[0,T\right], \end{array}$$

The existence of the solution is unique. *T*_*α*_ is the “conformable fractional-order derivative,” a continuous function of 1 < *α* < 2 < *f*, *g*, *h* : *J* × *X*⟶*X*, and *X* is the Banach space.

## 2. Related Work

Nonlinear differential equations are widely used in the modeling of complex nonlinear physical phenomena in many fields, such as electronic networks, meteorology, signal processing, and engineering science [8]. Due to the complexity of practical physical problems, when the order of derivatives in nonlinear partial differential equations is extended from integers to fractions [9], the nonlinear fractional-order partial differential equations are derived, which can more accurately characterize materials and nonlinear physical processes with time-memory properties and genetic properties [10].

To address these issues, the paper presents in detail the definition of the conformable fractional-order calculus, the integral, and the linearity properties under this definition, Rolle's theorem, and the mean value theorem [11]. A series of computational properties on the formable fractional-order calculus are given in [12], which include superposition of differential integrals, chain gauge, Gronwall's inequality, Taylor expansion, Laplace transform, and so on. The Taylor expansion of the conformable fractional-order calculus and its fractional-order Hayashi–Steffensen inequality, Hermite–Hadamard inequality, Chebyshev inequality, Ostrowski inequality, Jensen inequality, and 11 inequalities were proved in [13]. In addition, there are many studies on the properties of fractional-order calculus, which fully illustrate that the formable fractional-order calculus has very good properties [14, 15].

The method of partial integration is an important and fundamental class of methods for calculating integrals in calculus. It is derived from the multiplication rule of differentiation and the fundamental theorem of calculus. The common divisional integrals are organized in the order of divisional integrals according to the types of basic functions that make up the product function as a mnemonic: “against the power refers to three.” They refer to five types of basic functions: inverse trigonometric functions, logarithmic functions, power functions, exponential functions, and integrals of trigonometric functions, respectively.

In the last six years, research on conformable fractional-order calculus has made great progress: Shrauner in [16] explored two classes of conformable linear differential equations:

(3) $$\begin{array}{c} \left\{\begin{array}{c} T_{\alpha }^{a}y\left(t\right)+\frac{1}{a^{\alpha }}y\left(t\right)=g\left(t\right),\;t\in \left[a,b\right],\;a>0,\\ y\left(a\right)=y_{0}, \end{array}\right.\\ \left\{\begin{array}{c} T_{\alpha }^{a}y\left(t\right)+p\left(t\right)y\left(t\right)=g\left(t\right),\;t\in \left[a,b\right],\;a>0,\\ y\left(a\right)=y_{0}. \end{array}\right. \end{array}$$

Choi et al. [17] proved the sequential linear conformable fractional-order differential equation:

(4) $$\begin{array}{c} T_{n\alpha }y+p_{n-1}\left(t\right)T_{\left(n-1\right)\alpha }y+\cdots +p_{2}\left(t\right)T_{2\alpha }y+p_{1}\left(t\right)T_{\alpha }y+p_{0}\left(t\right)y=0,\\ T_{n\alpha }y+p_{n-1}\left(t\right)T_{\left(n-1\right)\alpha }y+\cdots +p_{2}\left(t\right)T_{2\alpha }y+p_{1}\left(t\right)T_{\alpha }y+p_{0}\left(t\right)y=q\left(t\right). \end{array}$$

(5) $$\begin{array}{c} T_{n\alpha }y+p_{n-1}T_{\left(n-1\right)\alpha }y+\cdots +p_{2}T_{2\alpha }y+p_{1}T_{\alpha }y+p_{0}y=0,\\ T_{n\alpha }y+p_{n-1}T_{\left(n-1\right)\alpha }y+\cdots +p_{2}T_{2\alpha }y+p_{1}T_{\alpha }y+p_{0}y=q\left(t\right), \end{array}$$

The above findings were all obtained for the case 0 < *α* ≤ 1. When *α* > 1, corresponding studies and analyses have also been done.

Akinyemi et al. [18] extended the above conclusions and studied the existence of positive solutions to the following conformable fractional-order edge value problem:

(6) $$\begin{array}{c} \left\{\begin{array}{cc} T_{\alpha }y\left(t\right)+f\left(t,y\left(t\right)\right)=0, & t\in \left[0,1\right],\\ y\left(0\right)=0, & y\left(1\right)=\lambda \int_{0}^{\eta }y\left(t\right)\text{d}t, \end{array}\right. \end{array}$$

where *α* ∈ (1,2], *η* ∈ (0,1], *f* : [0,1] × (0, *∞*]⟶(0, *∞*], and *λ* is the normal number.

## 3. Preliminary

The basic concepts and lemmas used in the article are as follows.

### 3.1. Conformable Fractional-Order Calculus

**Definition 1 .**

Let *α* ∈ (*n*, *n*+1], such that *β*=*α* − *n*; for a given function *f*, *g* : [*α*, +*∞*]⟶*ℜ*, if *f*(*n*) exists, then the conformable left derivative of *f* is defined as

(7) $$\begin{array}{c} T_{\alpha }^{a}f\left(t\right)=T_{\beta }^{a}f^{\left(n\right)}\left(t\right). \end{array}$$

Similarly, the conformable fractional-order right derivative of *f* is defined as

(8) $$\begin{array}{c} T_{\alpha }^{b}f\left(t\right)={\left(-1\right)}^{n+1}\left(T_{\beta }^{ba}f^{\left(n\right)}\right)\left(t\right). \end{array}$$

**Definition 2 .**

Let *α* ∈ (0,1]; then, the conformable fractional-order left integral of *f* is defined as

(9) $$\begin{array}{c} I_{\alpha }^{a}f\left(t\right)=\int_{a}^{t}f\left(x\right)\text{d}\alpha \left(x,a\right)\\ =\int_{a}^{t}{\left(x-a\right)}^{\alpha -1}f\left(x\right)\text{d}x. \end{array}$$

Similarly, the conformable fractional-order right integral of *f* is defined as

(10) $$\begin{array}{c} I_{\alpha }^{a}f\left(t\right)=\int_{a}^{t}f\left(x\right)\text{d}\alpha \left(x,a\right)\\ =\int_{a}^{t}{\left(x-a\right)}^{\alpha -1}f\left(x\right)\text{d}x, \end{array}$$

where *dα*(*b*, *x*)=(*b* − *x*)^*α*−1^*dx*.

### 3.2. Properties of the Conformable Fractional-Order Calculus

**Property 1 .**

If *f*(*a*)=*f*(*b*) : [*a*, *b*]⟶*ℜ*.*c* ∈ (*a*, *b*) is differentiable at point *t*_0_ > 0 of order *a*, then *f* is continuous at point *t*_0_.

**Theorem 1 .**

(conformable fractional-order differential median theorem). Let *α* > 0, and *f* : [*a*, *b*]⟶*ℜ*.∀*t* > *a* be satisfied:

1. *f* is continuous on [*a*, *b*].
2. *f* is *a*-order differentiable, where *α* ∈ (0, 1).

Then, there exists *c* ∈ (*a*, *b*) such that *T*_*α*_^*a*^*f*(*c*)=(*f*(*b*) − *f*(*a*)/(1/*α*)*b*^*α*^ − (1/*α*)*a*^*α*^).

**Theorem 2 .**

Let *f* : [*a*, +*∞*]⟶*ℜα* ∈ (*n*, *n*+1] be continuous and 0 < *α* ≤ 1; then, ∀*t* > *a*, *T*_*α*_^*a*^*I*_*α*_^*a*^*f*(*t*)=*f*(*t*).

**Definition 3 .**

Let *E*_1_ and *E*_2_ be two Banach spaces, ‖*m*‖_*L*^*P*^(*J*, *R*)_=() < *∞* : =sup{‖*u*‖ : *t* ∈ *J*}*L*^*P*^(*J*, *R*). Let the operator *A* : *D*⟶*E*_2_; if *A* maps any bounded set *S* in *D* to a column-tight set *A*(*S*) in *E*_2_ (i.e., *A*(*S*) is relatively tight, i.e., its closure *A*(*S*) is a tight set in *E*_2_), then *A* is said to be a tight operator that maps *D* into *E*_2_.

**Definition 4 .**

Let *E*_1_ and *E*_2_ be two Banach spaces, *D*⊆*E*_1_. Let the operator *A* : *D*⟶*E*_2_. If the operator *A* is continuous and tight, then *A* is a fully continuous operator that maps *D* into *E*_2_.

## 4. Solution Method

### 4.1. Invariant Subspace Method

Consider the subspace *W*_3_=*L*{1, *x*, *x*^2^} , whereupon an exact solution of the following form is obtained:

(11) $$\begin{array}{c} u\left(x,t\right)=C_{1}\left(t\right)+C_{2}\left(t\right)x+C_{3}\left(t\right)x^{2}, \end{array}$$

where *C*_1_(*t*), *C*_2_(*t*), *C*_3_(*t*) are the functions to be determined. Substituting (11), let all coefficients of the same power of *x* be equal to zero:

(12) $$\begin{array}{c} \frac{{\text{d}}^{\alpha }C_{1}\left(t\right)}{\text{d}t^{\alpha }}=C_{2}^{2}\left(t\right)+2C_{1}\left(t\right)C_{3}\left(t\right), \end{array}$$

(13) $$\begin{array}{c} \frac{{\text{d}}^{\alpha }C_{2}\left(t\right)}{\text{d}t^{\alpha }}=6C_{2}\left(t\right)C_{3}\left(t\right), \end{array}$$

(14) $$\begin{array}{c} \frac{{\text{d}}^{\alpha }C_{3}\left(t\right)}{\text{d}t^{\alpha }}=6C_{3}^{2}\left(t\right). \end{array}$$

Solving the system of equation (13) yields

(15) $$\begin{array}{c} C_{1}\left(t\right)=\frac{3a^{2}}{2}\frac{\Gamma \left(1-2\alpha \right)}{\Gamma \left(1-\alpha \right)}t^{-\alpha },\\ C_{2}\left(t\right)=at^{-\alpha },\\ C_{3}\left(t\right)=\frac{1}{6}\frac{\Gamma \left(1-\alpha \right)}{\Gamma \left(1-2\alpha \right)}t^{-\alpha }. \end{array}$$

An exact solution of (11) can be obtained as

(16) $$\begin{array}{c} u\left(x,t\right)=\frac{3a^{2}}{2}\left(\frac{\Gamma \left(1-\alpha \right)}{\Gamma \left(1-\alpha \right)}\right)t^{-\alpha }+axt^{-\alpha }+\frac{1}{6}\frac{\Gamma \left(1-\alpha \right)}{\Gamma \left(1-\alpha \right)}x^{2}t^{-\alpha }, \end{array}$$

where *α* is an arbitrary constant and *α* ∈ (0, (1/2)) ∪ ((1/2), 1).

### 4.2. Combination of Variable Separation and Chi-Square Method

Suppose that (11) has a solution of the following form:

(17) $$\begin{array}{c} u\left(x,t\right)=\sum_{k=0}^{m}a_{k}t^{\gamma k}x^{k}. \end{array}$$

By substituting (16) into the time fractional-order differential (11), it is easy to know that the highest number of *x* in *∂*^*α*^*u*/*∂t*^*α*^ is *m*, and the highest number of *x* in the nonlinear terms (*∂u*/*∂x*)^2^, *u*(*∂*^2^*u*/*∂x*^2^) is 2 *m*–2. Using the principle of chi-squared equilibrium, let *m*  = 2 *m*−2, and we can get *m*  = 2, so the exact solution of (11) has the following form:

(18) $$\begin{array}{c} u\left(x,t\right)=a_{0}t^{\gamma_{0}}+a_{1}t^{\gamma_{1}}x+a_{2}t^{\gamma_{2}}x^{2}, \end{array}$$

where *γ*_0_, *γ*_1_, *γ*_2_, *a*_0_, *a*_1_, *a*_2_ are constants to be determined. Substitute (17) into (11) to obtain

(19) $$\begin{array}{c} a_{0}\frac{\Gamma \left(\gamma_{0}+1\right)}{\Gamma \left(\gamma_{0}+1-\alpha \right)}t^{\gamma_{0}-\alpha }+a_{1}\frac{\Gamma \left(\gamma_{1}+1\right)}{\Gamma \left(\gamma_{1}+1-\alpha \right)}t^{\gamma_{1}-\alpha }x+a_{2}\frac{\Gamma \left(\gamma_{2}+1\right)}{\Gamma \left(\gamma_{2}+1-\alpha \right)}t^{\gamma_{2}-\alpha }x^{2}\\ =\left(a_{1}^{2}t^{2\gamma_{1}}+2a_{0}a_{2}t^{\gamma_{0}+\gamma_{2}}\right)+6a_{1}a_{2}t^{\gamma_{1}+\gamma_{2}}x+6a_{2}^{2}t^{2\gamma_{2}}x^{2}. \end{array}$$

In (18), let all powers of *t* be equal:

(20) $$\begin{array}{c} \gamma_{0}-\alpha =\gamma_{1}-\alpha =\gamma_{2}-\alpha =2\gamma_{1}=\gamma_{0}+\gamma_{2}=\gamma_{1}+\gamma_{2}=2\gamma_{2}. \end{array}$$

Solving (19) yields

(21) $$\begin{array}{c} \gamma_{0}=\gamma_{1}=\gamma_{2}=-\alpha . \end{array}$$

In (17), using the principle of chi-squared equilibrium, let

(22) $$\begin{array}{c} a_{0}\frac{\Gamma \left(\gamma_{0}+1\right)}{\Gamma \left(\gamma_{0}+1-\alpha \right)}=a_{1}^{2}+2a_{0}a_{2},a_{1}\frac{\Gamma \left(\gamma_{1}+1\right)}{\Gamma \left(\gamma_{1}+1-\alpha \right)}\\ =6a_{1}a_{2},a_{2}\frac{\Gamma \left(\gamma_{2}+1\right)}{\Gamma \left(\gamma_{2}+1-\alpha \right)}=6a_{2}^{2}. \end{array}$$

Solving (22) yields

(23) $$\begin{array}{c} a_{0}=\frac{3\Gamma \left(1-2\alpha \right)}{2\Gamma \left(1-\alpha \right)}a_{1}^{2},a_{1}=a_{1},a_{2}=\frac{\Gamma \left(1-\alpha \right)}{6\Gamma \left(1-\alpha \right)}. \end{array}$$

Substituting (21) and (23) into (17), an exact solution of (11) can be obtained as

(24) $$\begin{array}{c} u\left(x,t\right)=\frac{3\Gamma \left(1-2\alpha \right)}{2\Gamma \left(1-\alpha \right)}a_{1}^{2}t^{-\alpha }+a_{1}t^{-\alpha }x+\frac{\Gamma \left(1-\alpha \right)}{6\Gamma \left(1-2\alpha \right)}t^{-\alpha }x^{2}, \end{array}$$

where *a*_1_ is an arbitrary constant.

### 4.3. Combination of the Flush Equilibrium and Integral Branching Methods

(1) Assimilation refers to the transformation of acquired information so that it conforms to existing cognitive styles, although this transformation may distort the information to some extent. (2) Conformity refers to the alteration and adaptation of the conceptual model of the old knowledge to accommodate the new content after the child has acquired the new knowledge. (3) Balancing refers to a dynamic process of knowledge recognition that aims at a better state of equilibrium and generally occurs when the old and new information are evenly matched and one side cannot completely consume the other [19–22].

Assume that (11) has exact solutions of the following separated variable types.

(25) $$\begin{array}{c} u\left(x,t\right)=\left[a_{0}+a_{1}v\left(x\right)\right]t^{\gamma }. \end{array}$$

Substituting (24) into (11) yields

(26) $$\begin{array}{c} \frac{\Gamma \left(1+\gamma \right)}{\Gamma \left(1+\gamma -\alpha \right)}\left(a_{0}+a_{1}v\right)t^{\gamma^{\gamma -\alpha }}=\left[a_{1}^{2}{\left(\frac{\text{d}v}{\text{d}x}\right)}^{2}+\left(a_{0}a_{1}+a_{1}^{2}v\right)\frac{{\text{d}}^{2}v}{\text{d}x^{2}}\right]t^{2\gamma }. \end{array}$$

By the principle of chi-square equilibrium, let all the powers of *t* in (25) be equal:

(27) $$\begin{array}{c} \gamma -\alpha =2\gamma . \end{array}$$

The solution is *γ*=−*α*, which can be obtained by substituting (26) and eliminating *t*^−2*α*^.

(28) $$\begin{array}{c} \left(a_{0}a_{1}+a_{1}^{2}v\right)\frac{{\text{d}}^{2}v}{\text{d}x^{2}}+a_{1}^{2}{\left(\frac{\text{d}v}{\text{d}x}\right)}^{2}-a_{1}\Omega_{0}v-a_{0}\Omega_{0}=0, \end{array}$$

where Ω_0_=(Γ(1 − *α*)/Γ(1 − 2*α*)), such that d*v*/d*x*=*y*. (34) can be reduced to the following singular planar dynamical system:

(29) $$\begin{array}{c} \left\{\begin{array}{c} \frac{\text{d}v}{\text{d}x}=y,\\ \frac{\text{d}y}{\text{d}x}=\frac{\left(a_{0}\Omega_{0}/a_{1}\right)+\Omega_{0}v-a_{1}y^{2}}{a_{0}+a_{1}v}. \end{array}\right. \end{array}$$

It is easy to find that when *v*=−(*a*_0_/*a*_1_), d*y*/d*x* is meaningless and systems (28) and (29) are not equivalent. System (29) is not equivalent to (28), and *v*=−(*a*_0_/*a*_1_) is a nontrivial solution of (28). In order to obtain a system that is completely equivalent to (28) no matter how the function *v* varies, the following transformation is required:

(30) $$\begin{array}{c} dx=\left(a_{0}+a_{1}v\right)\text{d}\tau , \end{array}$$

where *τ* is a parameter, so that system (29) can be reduced to a regular planar system:

(31) $$\begin{array}{c} dx=\left(\left\{\begin{array}{c} \frac{\text{d}v}{\text{d}\tau }=\left(a_{0}+a_{1}v\right)y,\\ \frac{\text{d}y}{\text{d}\tau }=\frac{a_{0}\Omega_{0}}{a_{1}}+\Omega_{0}v-a_{1}y^{2}. \end{array}\right.\right. \end{array}$$

Obviously, systems (29) and (31) have the same first integral:

(32) $$\begin{array}{c} y^{2}=\frac{\left(2\Omega_{0}/3a_{1}^{2}\right){\left(a_{0}+a_{1}v\right)}^{3}+h}{{\left(a_{0}+a_{1}v\right)}^{2}}, \end{array}$$

where *h* is a constant of integration. (32) can be rewritten as

(33) $$\begin{array}{c} H\left(v,y\right)\equiv {\left(a_{0}+a_{1}v\right)}^{2}y^{2}-\frac{2\Omega_{0}}{3a_{1}^{2}}{\left(a_{0}+a_{1}v\right)}^{3}=h. \end{array}$$

Obviously, system (32) has only one equilibrium point *P*(−(*a*_0_/*a*_1_), 0) on the *v*-axis and *H*(−(*a*_0_/*a*_1_), 0)=0. In fact, when *h*=*H*(−(*a*_0_/*a*_1_), 0)=0, it is easy to obtain the solution *v*(*x*) of (31).

### 4.4. The Separation of Function Variable Method and the Separation of Generalized Variables by the Airy Equation Method

**Case 1 .**

Application of the method of separation of functional variables [23, 24].

Suppose the solution of (34) has the following form:

(34) $$\begin{array}{c} u=F\left(z\right),z=mx+\psi \left(t\right), \end{array}$$

where *F*(*z*), *ψ*(*t*) are the unknown functions to be determined. Plugging (35) into (34) yields the following generalized differential equation:

(35) $$\begin{array}{c} t^{1}-\alpha F^{\prime }\psi^{\prime }+m^{3}F^{\prime \prime }=0. \end{array}$$

For some constants *μ*, we have

(36) $$\begin{array}{c} F^{\prime }=m^{3}\mu F^{\prime \prime }, \end{array}$$

and

(37) $$\begin{array}{c} -\mu t^{1-\alpha }\psi^{\prime }=1. \end{array}$$

Solving (36) and (37), we have the following.

(1) Type 1: when *μ* > 0, then
  (38) $$\begin{array}{c} F\left(z\right)=C_{1}+C_{2}e^{\left(1/\sqrt{m^{3}\mu }\right)z}+C_{3}e^{-\left(1/\sqrt{m^{3}\mu }\right)z}. \end{array}$$
(2) Type 2: when *μ* < 0, then
  (39) $$\begin{array}{c} F\left(z\right)=C_{1}+C_{2}\cos\frac{1}{\sqrt{-m^{3}\mu }}z+C_{3}\sin\frac{1}{\sqrt{-m^{3}\mu }}z, \end{array}$$
  and
  (40) $$\begin{array}{c} \psi \left(t\right)=-\frac{t^{\alpha }}{\mu \alpha }+C_{4}, \end{array}$$
  where *C*_*i*_(*i*=1,…, 4) is an arbitrary constant and is a nonzero constant. Combining equations (38), (39), and (40), the following two traveling wave solutions are obtained:
  (41) $$\begin{array}{c} u_{1}\left(x,t\right)=C_{1}+C_{2}\exp\left\{\frac{1}{\sqrt{m^{3}\mu }}\left(mx-\frac{t^{\alpha }}{\mu \alpha }+C_{1}\right)\right\}+C_{3}\exp\left\{-\frac{1}{\sqrt{m^{3}\mu }}\left(mx-\frac{t^{\alpha }}{\mu \alpha }+C_{4}\right)\right\}, \end{array}$$
  and
  (42) $$\begin{array}{c} u_{2}\left(x,t\right)=C_{1}+C_{2}\cos\frac{1}{\sqrt{-m^{3}\mu }}\left(mx-\frac{t^{\alpha }}{\mu \alpha }+C_{4}\right)+C_{3}\sin\frac{1}{\sqrt{-m^{3}\mu }}\left(mx-\frac{t^{\alpha }}{\mu \alpha }+C_{4}\right). \end{array}$$

With the help of Maple software, if we take *C*_1_=*C*_4_=1, *C*_2_=2, *C*_3_=3, *μ*=−1, *α*=0.7 in (42), we can derive the 3D figure of *u*_2_(*x*, *t*), as shown in Figure 1. (2 and 3).

**Case 2 .**

Application of the generalized variable separation method.

(1) Assumptions:
  (43) $$\begin{array}{c} \left\{\begin{array}{c} \varphi \left(x\right)=-\frac{\mu }{6}x^{3}+C_{1}x^{2}+C_{2}x+C_{3},\\ \psi \left(t\right)=\frac{\mu t^{\alpha }}{\alpha }+C_{4}. \end{array}\right. \end{array}$$
(2) Substituting (43) into (34), we get
  (44) $$\begin{array}{c} \varphi \left(x\right)t^{1-\alpha }\psi^{\prime }\left(t\right)+\varphi^{\prime \prime }\left(x\right)\psi \left(t\right)=0. \end{array}$$
(3) For some constants *μ*, we have
  (45) $$\begin{array}{c} u_{5}\left(x,t\right)=-\frac{\mu }{6}x^{3}+C_{1}x^{2}+C_{2}x+\frac{\mu t^{\alpha }}{\alpha }+C_{3}+C_{4}, \end{array}$$
  and
  (46) $$\begin{array}{c} \varphi^{\prime \prime }\left(x\right)+\mu \varphi \left(x\right)=0. \end{array}$$
(4) Solving (45) and (46), we have the following.
  (1) Type 1: when *μ* > 0, then
    (47) $$\begin{array}{c} \varphi \left(x\right)=C_{1}e^{\sqrt[{3}]{-\mu }x}+\frac{e^{\sqrt[{3}]{\mu }x}}{2}\left(C_{2}\cos\left(\frac{\sqrt{3}\sqrt[{3}]{\mu }x}{2}\right)+C_{3}\sin\left(\frac{\sqrt{3}\sqrt[{3}]{\mu }x}{2}\right)\right). \end{array}$$
  (2) Type 2: when *μ* < 0, then
    (48) $$\begin{array}{c} \varphi \left(x\right)=C_{1}e^{\sqrt[{3}]{-\mu }x}+\frac{e^{\sqrt[{3}]{\mu }x}}{2}\left(-C_{2}\sin\left(\frac{\sqrt{3}\sqrt[{3}]{-\mu }x}{2}\right)+C_{3}\cos\left(\frac{\sqrt{3}\sqrt[{3}]{-\mu }x}{2}\right)\right), \end{array}$$
    and
    (49) $$\begin{array}{c} \psi \left(t\right)=C_{4}e^{\mu t^{\alpha }\alpha /\alpha }, \end{array}$$
    where *C*_*i*_(*i*=1,…, 4) is an arbitrary constant and *C*_4_ is a nonzero constant. In conclusion, combining equations (47)–(49) and (45), the exact solution is obtained. (34) has the following form:
    (50) $$\begin{array}{c} u_{3}\left(x,t\right)=C_{4}e^{\mu t^{\alpha }/\alpha }\left(C_{1}e^{\sqrt[{3}]{-\mu }x}+\frac{e^{\sqrt[{3}]{\mu }x}}{2}\left(C_{2}\cos\left(\frac{\sqrt{3}\sqrt[{3}]{\mu }x}{2}\right)+C_{3}\sin\left(\frac{\sqrt{3}\sqrt[{3}]{\mu }x}{2}\right)\right)\right), \end{array}$$
    and
    (51) $$\begin{array}{c} u_{4}\left(x,t\right)=C_{4}e^{\mu t^{\alpha }/\alpha }\left(C_{1}e^{\sqrt[{3}]{-\mu }x}+\frac{e^{\sqrt[{3}]{\mu }x}}{2}\left(-C_{2}\sin\left(\frac{\sqrt{3}\sqrt[{3}]{\mu }x}{2}\right)+C_{3}\cos\left(\frac{\sqrt{3}\sqrt[{3}]{\mu }x}{2}\right)\right)\right). \end{array}$$
(5) With the help of Maple software, if we take *C*_1_=1, *C*_2_=2, *C*_3_=*C*_4_=0, *μ*=5, *α*=0.9 in (50), we can derive the 3D figure of *u*_3_(*x*, *t*). If we take *C*_1_=*C*_4_=1, *C*_2_=2, *C*_3_=3, *μ*=−1, *α*=0.7, we can obtain the 3D figure of *u*_4_(*x*, *t*), as shown in Figure 2.
(6) Assumptions:
  (52) $$\begin{array}{c} u\left(x,t\right)=\varphi \left(x\right)+\psi \left(t\right),\left(\varphi \left(x\right)\neq 0,\psi \left(t\right)\neq 0\right). \end{array}$$
(7) Substituting (52) into (34), we get
  (53) $$\begin{array}{c} t^{1-\alpha }-\mu \psi^{\prime }\left(t\right)+\varphi^{\prime \prime }\left(x\right)=0. \end{array}$$
(8) For some constants *μ*, we have
  (54) $$\begin{array}{c} t^{1-\alpha }-\mu \psi^{\prime }\left(t\right)=\mu , \end{array}$$
  and
  (55) $$\begin{array}{c} -\varphi^{\prime \prime }\left(x\right)=\mu . \end{array}$$
(9) Solving equations (54) and (55), we obtain
  (56) $$\begin{array}{c} \left\{\begin{array}{c} \varphi \left(x\right)=-\frac{\mu }{6}x^{3}+C_{1}x^{2}+C_{2}x+C_{3},\\ \psi \left(t\right)=\frac{\mu t^{\alpha }}{\alpha }+C_{4}, \end{array}\right. \end{array}$$
  where *C*_*i*_(*i*=1,…, 4) are arbitrary constants. With the help of (56) and (53), we obtain the exact solution of (34) in the following form:
  (57) $$\begin{array}{c} u_{5}\left(x,t\right)=-\frac{\mu }{6}x^{3}+C_{1}x^{2}+C_{2}x+\frac{\mu t^{\alpha }}{\alpha }+C_{3}+C_{4}. \end{array}$$
(10) With the help of Maple software, if we take *C*_1_=1, *C*_2_=2, *C*_3_=*C*_4_=0, *μ*=5, *α*=0.9 in (57), we can derive the 3D figure of *u*_5_(*x*, *t*) as shown in Figure 3.

## 5. Conclusion

The significant advantage of fractional-order mathematical models over integer-order integral is that they can better simulate various physical phenomena in science and technology and have a deep physical background. In addition, we also obtained a series of physical breakwaters, selected some of them using MAPL, and displayed their 3D images. In addition, we observe that such a simple and easy method is an effective method, which can be used to solve fractional compatible differential equations.

## Figures and Tables

**Figure 1:** 3D diagram of *u*_2_(*x*, *t*).

**Figure 2:** 3D diagram of *u*_3_(*x*, *t*) and *u*_4_(*x*, *t*).

**Figure 3:** 3D diagram of *u*_5_(*x*, *t*).

## Data Availability

The experimental data used to support the findings of this study are available from the corresponding author upon request.
